This article has been retracted.

# Ageing Design of Urban Park Landscape Based on Computer Virtual Simulation Technology

**DOI:** 10.1155/2022/3150371

**Published:** 2022-07-31

**Authors:** Jing Fan

**Affiliations:** School of Art Design, Xi'an FanYi University, Xi'an 710105, Shaanxi, China

## Abstract

Greenery are the parks in the urban areas and it becomes progressively most significant as cities grow more crowded. In the end, urban parks contribute to the population's healthiness and welfare by providing opportunities intended for physical and social activity, leisure, and relaxation. In order to construct “Digital Land,” computer and system software and hardware were used. Computer simulations are used to examine the value of a city garden's landscape design. Digital models and multimedia performances are being built using computer-aided design (CAD), this underlines the need for digitizing data for landscape design. A region's landscapes can only be accurately assessed if sufficient information is available on the elements that influence the people's awareness of landscape quality, as well as the kind, method, and effective rate of each of them. We use an LVQANN (artificial neural network) to forecast the landscape aesthetic assessment of urban parks and priorities the model's significant factors in this research. User viewpoint and artificial neural network modelling were utilized in conjunction to assess the aesthetic quality of the urban park's environment. This was done for two reasons. The design of urban parks decision support system is known as MATLAB software's multilayer perceptions model, which gives the ability to anticipate landscape visual significance in innovative parks. In this study, the ANN LVQ model is used to execute an ageing design of an urban park landscape based on a computer virtual simulation application. An example land is selected as input and area linked to sunny spot, top view, and so on is fixed. The ANN tool box is used to develop this application in MATLAB 2018b software. The following approach is used to create the ideal urban park landscape model. An accuracy of 89.23 percent, a sensitivity of 87.34 percent, and a recall of 78.93 percent were achieved, outperforming the approach and competing with the current model.

## 1. Introduction

For inhabitants, urban parks provide low-cost chances to connect with nature in their everyday lives, while also improving the aesthetics of the city. In order to accurately analyze a region's landscapes, it is necessary to know the kind, method, and effect rate of each of the influential aspects, as well as how they affect the user's sense of landscape quality. Environmental, biological, social, cultural, and physiological aspects all have a role in landscape's aesthetic value. For the majority of individuals, landscape variety, kind of landscape, and people's taste and ideals all play a role in aesthetic choice.

Designing Tehran's urban parks now adheres to the guidelines outlined in Vice President for Strategic Planning and Supervision publication No. 203, with some minor modifications. This has resulted in a dramatic decrease in the park's landscape structure's aesthetic value, and there is no specific framework for increasing landscape quality. Which landscape aspects are most appealing to users and which are the most important variables in influencing their view of the environment? How can we forecast the aesthetic worth of urban parks in the eyes of observers by constructing the most suitable structure? ‘The factors that affect the aesthetic quality of natural surroundings were found to be the viewpoint, land slope, and landform. Researchers feel that assessing the visual excellence of a land and its ecosystem requires paying close attention to the physical conditions of the landscape (which is illustrated in Figure 1).

This has looked at the role that water plays in enhancing the aesthetics of the park and drawing in more visitors. Water features like ponds, pools, runnels, fountains, etc., should be included into landscape design, says one researcher, in order to provide park visitors with more diversity and enjoyment. For the evaluation of urban green space, Jahani and Mohammadi Fazel employed CNN modelling to determine characteristics and indications such as bared surfaces, architectural features, water, trees and shrubs, sports equipment, and mountain vistas as beneficial landscape beautifying aspects. Landscapes are classed as high-quality if they offer access to water, leisure, and sports equipment, according to studies. In addition to trees and plants, architecturally appealing buildings, and mountain vistas, urban green space has a better landscape quality. With the introduction of a multilayer perception model, the diversity of tree species and pure natural regions devoid of human interventions such as buildings, paths, and park equipment were given a boost in the landscape quality of natural areas. It is possible to utilize any of the design concepts outlined in these studies as indications of the current research as shown in Figure 1.

The contribution of the work is as follows:

- To execute an ageing design of an urban park landscape by using the ANN LVQ model based on a computer virtual simulation application.
- To select the example land and taking it as an input and area linked to sunny spot, top view, and so on is fixed and perform evaluation.

### 1.1. Literature Survey

Jo and Jeon consider the relevance of human components; we determined that designs are required to encourage an adequate degree of park-goers to boost their overall contentment with the surroundings. An urban park setting may be made more enjoyable by using this study's results as design recommendations and supporting data [1].

Yu et al. As a result of using ArcGIS 3-D analysis, we want to present a novel study viewpoint and a service that provides techniques for creating layouts of such places that are beneficial for the elderly in order to better assure urban sustainability civilization [2].

Li and Xu Moreover, the research study and effectiveness test results show that the realized distribution rationality technology is better than the competition. This method might serve as a scientific reference and basis for the present landscape gardening industry to include 3-D images and other cutting-edge technologies [3].

Van Vliet et al. In an urban park, the natural components and a wide range of floral species are vital while the services provided vary widely in value among various sectors of the public Research like this might help park planners and legislators make better choices. As a result, it shows the value of establishing a virtual park in environmental preference study. Check out the full-length article [4].

Luo and Liu. As the rehabilitation environment evolves, this study examines present empirical research methodologies from the perspectives of subject and object, pointing out their flaws, forecasting their future development trends, and ultimately proposing future empirical research. The study should be more rigorous and methodical, with a better knowledge of what the research is about, and the establishment of an assessment system with the most practical significance possible should be encouraged [5].

Yang The urban parks landscape design and analysis of city parks significance may be improved by using computer simulation. More and more people are realising how important digitising information is to creating digital models and multimedia performances in computer-aided design (CAD), particularly when it comes to the landscape design process [6].

Ma et al. Analyzing the garden's rational distribution is based on a new three-dimensional picture. Virtual reality technology was used to build a three-dimensional simulation of the distribution landscape's efficacy. Finally, the garden, rational medication delivery methods, case studies, benefits, and results of performance tests will be discussed [7].

Irvine et al. To better understand the challenges of combining multidisciplinary visioning and modelling of green space design and performance evaluation in the Thai town of Cha Am, we interviewed students from three universities: Thammasat University, Mahidol University, and AIT. Examples from Phnom Penh illustrate how 3D visualisation and modelling might help people better comprehend the benefits of green space. For urban green space design to be successful, we believe that a decision support system that is easy to use is essential [8].

Bishop and Rohrmann findings from the study suggest that the most meticulous and time-consuming computer simulations may not always reflect actual-world behaviour. However, the realism evaluations of the viewers were largely positive, and the contrasts between day and night circumstances in the simulated environment are almost identical to those in the actual world. The results reveal areas in need of improvement and reassessment [9].

Jeon and Hong. Various human activities in parks have been shown to have a significant effect in influencing soundscape perception. There was also a strong link between how people perceived soundscapes and the aesthetic quality, simplicity, and feeling of enclosure provided by a given environment. As a consequence of this study, soundscapes in urban parks might benefit from the findings, even if they are only applicable to Seoul's specific settings [10].

Daniel and Meitner. Each degree of realism–abstraction was used to portray the identical woodland landscape images in this investigation. One similar set of forest landscape images was given to various groups of observers, and each group was asked to score the perceived scenic quality of the scenes. Computer-generated landscape visualisations may not be accurate representations of the landscape since correlations between judgments of the same landscapes in various visualisation situations were very low [11].

Lange. This investigation focuses on the subject of whether, how, and to what extent virtual landscapes can be used to accurately reproduce genuine landscapes seen in images. The settlements of Schwyz and Ingenbohl–Brunnen, located on the shores of Lake Lucerne in Central Switzerland, are the focus of this research [12].

Bishop and Lange. The field of visualisation technology has a lot to offer, and notable developers discuss the latest advancements in hardware, software, and display technology. Concerns about the legitimacy and ethics of the use of visual simulations are raised. Authors from forestry, agriculture, mining, energy, and urban planning have contributed cutting-edge applications. Finally, a look at what's to come in terms of augmented reality and public engagement is included in the volume's last chapter [13].

Bishop. The view analysis of Two-Dimensional GIS's approach is ineffective in circumstances when significant 3D aspects are present. For landscape visual interpretation, a new standard is required due to an increase in agent-based modelling. Both GIS-based visual modelling and 3D-based visual modelling are examined in this paper [14].

Thompson It is suggested that open space be defined and used in a more flexible manner, taking into account ‘loose-fit' landscapes that provide possibilities for the socially marginalised and environmentally moving within a dynamic context of urban structures and networks [15].

Wergles and Muhar. Visualizations, on the other hand, were more effective in conveying particular features of the design because of their capacity to draw the viewer's attention to focal points. As a means of conveying design concepts, visual representations may work well, but they must be tailored to the audience in order to be effective [16].

Sheppard Ethical and scientific validity may be improved by providing direction and assistance to visualisation practitioners, according to a suggested framework. An preliminary code of ethics is offered for evaluation, testing, and change by other researchers and users until more thorough results are gathered from the vast amount of study required on this topic. Such a code should incorporate general principles and guidelines for ethical behaviour in the creation, presentation, and analysis of visualisations, as well as the analysis of user comments [17].

Appleton and Lovett. According to the data, it seems that certain characteristics are more significant than others when it comes to realism. Ratings were significantly influenced by foreground vegetation and the general appearance of the ground surface, despite a large variation in ratings across the three situations evaluated [18].

Kort et al. On four measures, researchers discovered substantial variations. Environment and plants, on the other hand, did not seem to interact in a major way. Virtual environments have many characteristics with actual ones, but there are also significant distinctions. As a result, we believe that this is an important and fascinating topic for environmental psychology [19].

Orland et al. Using virtual reality (VR) technology to aid with environmental decision-making is the focus of this article. Human-computer interfaces are discussed and categorized, and then we examine how VR's qualities match up with landscape representation demands [20].

The drawback of the existing approaches is as follows, expensive direct observations, it requires numerous employs for monitoring the extended periods and restricted information only provided.

## 2. Methodology

In this section, urban park landscape-based analysis was performed using LVQ ANN technology. For multiclass classification, LVQ (learning vector quantization) is a prominent class of adaptable nearest prototypes classifiers. However, learning algorithms from this family have been developed on heuristic grounds so far. LVQ (Learning Vector Quantization) classifiers are reviewed in this article. A suggested taxonomy incorporates the most significant LVQ techniques to date. The fundamental elements of contemporary LVQ techniques are outlined in this article. 11- LVQ extractors are compared by means of a real-world dataset and 2 fake areas shown in Figure 2.

(1) $$\begin{array}{c} y=\left\{y\left(t\right)|t=o,1,2,\ldots d-1\right\}. \end{array}$$

Here, the quantity of Urban park area [5] for time. *t*, *d*: length of network traffic duration.

The domain represents a discrete-time series of finite length *according* to ANN theory. So,

(2) $$\begin{array}{c} x\left(n\right)=y\left(t\right),n=t,n=0,1,\ldots ,d-1. \end{array}$$

This discrete series *x*(*n*) represents the set given below,

(3) $$\begin{array}{c} \left\{x\left(0\right)=y\left(1\right),x\left(1\right)=y\left(2\right),\ldots .x\left(d-1\right)=y\left(z\right)\right\}. \end{array}$$

The ANN *x*(*n*) with finite length *d* is considered as a sequence of periodic nature. Subsequently, with the theory of ANN.

(4) $$\begin{array}{c} X\left(k\right)=\overset{d-1}{\underset{n=0}{\sum }}\left(x\left(n\right)e^{-j\left(2\pi /d\right)nk}\right),\;0\leq k\leq d-1. \end{array}$$

Consequently, *x*(*n*) is expanded as the equation given below:

(5) $$\begin{array}{c} x\left(n\right)=\frac{1}{z}\overset{z-1}{\underset{k=0}{\sum }}\left(Y\left(k\right)e^{j\left(2\pi /d\right)nk}\right),\;0\leq n\leq d-1. \end{array}$$

From (2) and (5), the value of *y*(*t*) at time *t* is obtained as follows:

(6) $$\begin{array}{c} \tilde{y}\left(t\right)=y\left(n\right)=\frac{1}{z}\overset{z-1}{\underset{k=0}{\sum }}\left(Y\left(k\right)e^{j\left(2\pi /d\right)nk}\right),t=n,0\leq n\leq d-1. \end{array}$$

Since the network traffic considers *x*(*t*) ≥ 0, the equation below is attained for accessing traffic in network.

(7) $$\begin{array}{c} \left\{\begin{array}{c} \tilde{y}\left(t\right)=\frac{1}{z}\overset{z-1}{\underset{k=0}{\sum }}\left(Y\left(k\right)e^{j\left(2\pi /d\right)nk}\right),\;0\leq n\leq d-1,\\ \tilde{y}\left(t\right)\geq 0. \end{array}\right. \end{array}$$

Equation (7) represents that the traffic across network is extended to Fourier series with the duration length *d* as well as network traffic correlation at *d* − 1 time points. The Fourier series expansion matrix is given by the following:

(8) $$\begin{array}{c} \hat{y}=\left[\begin{array}{ccc} {\hat{y}}_{0,0} & {\hat{y}}_{0,1}\ldots .. & {\hat{y}}_{0,d-1}\\ {\hat{y}}_{1,0} & {\hat{y}}_{1,1}\ldots .. & {\hat{y}}_{1,d-1}\\ {\hat{y}}_{d-1,0} & {\hat{y}}_{d-1,1}\ldots .. & {\hat{y}}_{d-1,d-1} \end{array}\right]. \end{array}$$

Hence, we get the following:

(9) $$\begin{array}{c} \hat{y}={\left({\hat{y}}_{0},{\hat{y}}_{1},\ldots {\hat{y}}_{d-1}\right)}^{T}. \end{array}$$

Here, *T*: matrix transposition operation

(10) $$\begin{array}{c} \text{Consequently},\;{\hat{y}}_{i}=\left({\hat{y}}_{i,0},\ldots {\hat{y}}_{i,d-1}\right). \end{array}$$

In which, *i*=0,1,……., *d* − 1

From (7),

(11) $$\begin{array}{c} {\hat{y}}_{i,k}=X\left(k\right)e^{j\left(2\pi /d\right)ik}, \end{array}$$

where. *i*, *k*=0,1,….., *d* − 1

Here, (8) captures the relation within the network traffic effectively. Subsequently,

(12) $$\begin{array}{c} \hat{y}=UDV^{T},U,V,D\text{ and }V\text{ are}d\times d\text{ matrices}. \end{array}$$

*D* and *V* represent the network traffic features and equation (12) captures the area dimensions features.

(13) $$\begin{array}{c} K\left(d\right)=\frac{p_{0}}{2}+\overset{d}{\underset{k=1}{\sum }}\left(p_{k}\cos kx+q_{k}\sin kx\right). \end{array}$$

The authentication key for the time duration *d*+1 is given by,

(14) $$\begin{array}{c} K\left(d+1\right)=\frac{p_{0}}{2}+\overset{d+1}{\underset{k=1}{\sum }}\left(p_{k}\cos kx+q_{k}\sin kx\right), \end{array}$$

(15) $$\begin{array}{c} =K\left(d\right)+\left(p_{d+1}\cos\left(d+1\right)x+q_{d+1}\sin\left(d+1\right)x\right). \end{array}$$

The authentication key *K*(*d*+1) for time period *d*+1 is calculated by *K*(*d*) as well as the Fourier series coefficients *p*_*d*+1_ and *q*_*d*+1_.

In statistical classification and prediction, LVQ (Learning Vector Quantization) is a family of methods that try to learn prototypes (codebook vectors) that represent class areas. Voronoi partitions are used to define the class areas as hyperplanes between prototypes. Late in the '80s, Teuvo Kohonen came up with LVQ1 an algorithm that has since been used in many different ways. There has been a small but dedicated group of researchers studying LVQ algorithms since their introduction. “Learning Vector Quantization” or “LVQ” appeared in the titles or abstracts of 665 academic articles that were indexed by the ISI Web of Science in November 2013. This article presents a survey of recent developments in the subject.

In order to achieve competitive learning's, LVQ algorithms are similar to SOMs and c-means. During training, the winner-takes-all learning rule and variations based on iterative URBAN PARK _SCAPE_002ates to just selected components or neighborhoods are used to create competitive learning algorithms. Class-labeled prototypes are obtained via supervised learning in the original LVQ technique and most recent extensions (classifiers). Unsupervised learning may also be used to train LVQ for clustering without labels. We will exclusively cover LVQ classifiers in this work.

Data are supposed to have a Gaussian mixture probability density function (URBAN PARK _SCAPE_002f). Logarithmically maximizing the difference between the proper class's and erroneous class ‘URBAN PARK _SCAPE_002f ratios is a cost function given a data point.

In addition, GLVQ and the original LVQ algorithms have been improved in terms of their initialization sensitivity [15].

For example, LVQ may be used in image and signal processing, the biomedical area, and medicine and industry, just to mention a few examples of its many uses There is a vast collection of bibliographic data accessible in the system.

In this study, we give a thorough overview of the most significant supervised LVQ algorithms since Teuvo Kohonen's initial work. Our taxonomy and techniques for LVQ classification are presented here. A total of eleven different LVQ algorithms are tested on a variety of simulated and real-world datasets. Depending on the kind of datasets, we explore the benefits and drawbacks of each strategy.

Assuming that the input space contains a number of reference vectors *Wk*. Typically; a class is allocated a number of reference vectors. This means that input vector *x* has been assigned a classification based on the closest reference vector. We may think of *Wk* (*t*) as the discrete-time representation of *Wk* sequences. In this part, we will concentrate on LVQ2.1, which has been offered before. This is how LVQ2.1 URBAN PARK_SCAPE_002ates your reference vectors from a set of correctly specified beginning values.

(16) $$\begin{array}{c} \min\left(\frac{d_{i}}{d_{j}},\frac{d_{j}}{d_{i}},\right)>S. \end{array}$$

As in, di = Ix−*WD* and *d*_i_ = Ix−*WD* + wjl.

Based on the notion of pushing decision boundaries toward Bayesian bounds by applying attractive and repulsive pressures from *x*, LVQ2.1 implements an algorithmic approach (shown in Figure 3). As a result, the reference vectors diverge in the long term since no consideration is paid to the *Wk* location. Referencing the class distributions using multiple reference vectors has been suggested as a way of preventing reference vector divergence. However, LVQ3 has the same properties as the earlier LVQ2.1 and so does not address the issue of reference vector divergence.

## 3. Results and Discussion

In this section, a brief discussion of urban park landscapes are finding via the MATLAB-based ANN computer vision model.

The parameter estimation is shown in Table 1:

Figure 4 clearly explains about the top view model of a proposed design estimating image; in this, using ANN LVQ model attains proper landscape architecture.

Figure 5 clearly explains about different views of selected urban area, in this proposed green roof initiatives have been used to enhance climatic conditions, conserve and develop plant, encourage outdoor activities and active lifestyles, stimulate social connection and exchange, and create healthy urban circumstances for cognitive and emotional well-being.

Figure 6 clearly explains about the inner layout of urban park landscape analysis, in this all-road maps and paths are added accordingly.

Given the limited extent of these green spaces, design standards must be simple: trees, bushes, and grass areas must be placed in such a manner that shaded and sunny places alternate; paved areas must also be given, with areas for playing and relaxing shown in Figure 7.

The results' comparison is shown in Table 2:

Figure 8 clearly explains about different comparison of results of proposed model, in this proposed ANN_LVQ model attains more improvement. Functionality variation arises in the process of simulation, this system compares the sensitivity of the system with random variations and this results in the decrease of computational speed.

## 4. Conclusion

In this research work, ageing design of urban park landscape based on computer virtual simulation application is implemented using ANN LVQ model. The visual quality of 100 urban park settings was assessed using citizen perception. A total of 15 landscape characteristics impacted the visual quality of the scene. According to the findings, the multi-layer perceptions model 15-8-1 with a configuration of 15-8-1 (15 input variables, 8 hidden layer neurons, and 1 output variable) has the best structure optimization performance. Three data sets were obtained with R2 values of 0.97, 0.88, and 0.90: training (validation), test, and (test). The visual quality of urban park landscapes is most affected by land slope and vegetation/building/hard surface ratios with model sensitivity values of 0, 24, 0, 7, and 0. In this an example land is selecting as input and fixing area related to sunny place, top view etc. This application is implemented on MATLAB 2018b software using ANN tool box. The perfect urban park landscape model is designed using following technique. The measures like accuracy 89.23%, sensitivity 87.34% and recall 78.93% had been attained those are out performance the methodology and compete with present model.

## Figures and Tables

**Figure 1:** Urban park landscape.

**Figure 2:** Proposed block.

**Figure 3:** MATLAB-based ANN LVQ analysis.

**Figure 4:** Top view for selected urban park landscape.

**Figure 5:** Computer level design with ANN.

**Figure 6:** Inner layout.

**Figure 7:** Final layout.

**Figure 8:** Comparison of results.

**Table 1:** Parameter estimation.

Regression weights	Estimate	S.E.	C.R.	*P*
UP-1 <---URBAN PARK _SCAPE	1.000			
UP-2 <---URBAN PARK _SCAPE	1.440	0.149	9.675	^*∗∗∗*^
UP-3 <---URBAN PARK _SCAPE	1.733	0.161	10.778	^*∗∗∗*^
UP-4 <---URBAN PARK _SCAPE	1.894	0.174	10.875	^*∗∗∗*^
UP-5 <---URBAN PARK _SCAPE	1.458	0.144	10.141	^*∗∗∗*^
UP-6 <---URBAN PARK _SCAPE	1.246	0.126	9.886	^*∗∗∗*^
UP-7 <---URBAN PARK _SCAPE	1.723	0.147	11.700	^*∗∗∗*^
UP01-6 <---URBAN PARK _SCAPE_001	1.000			
UP01-5 <---URBAN PARK _SCAPE_001	3.596	1.396	2.576	0.010
UP01-4 <---URBAN PARK _SCAPE_001	4.129	1.584	2.607	0.009
UP01-3 <---URBAN PARK _SCAPE_001	4.297	1.648	2.607	0.009
UP01-2 <---URBAN PARK _SCAPE_001	0.721	0.491	1.469	0.142
UP01-1 <---URBAN PARK _SCAPE_001	1.403	0.631	2.223	0.026
URBAN PARK _SCAPE_002-6 <--- URBAN PARK	1.000			
URBAN PARK _SCAPE_002-5 <---URBAN PARK	0.911	0.116	7.883	^*∗∗∗*^
URBAN PARK _SCAPE_002-4 <---URBAN PARK	0.939	0.110	8.533	^*∗∗∗*^
URBAN PARK _SCAPE_002-3 <---URBAN PARK	1.151	0.122	9.441	^*∗∗∗*^
URBAN PARK _SCAPE_002-2 <---URBAN PARK	0.827	0.092	9.006	^*∗∗∗*^
URBAN PARK _SCAPE_002-1 <---URBAN PARK	1.042	0.105	9.954	^*∗∗∗*^
TAD-6 <---LANDSCAPE analysis	1.000			
TAD-5 <---LANDSCAPE analysis	1.208	0.139	8.662	^*∗∗∗*^
TAD-4 <---LANDSCAPE analysis	1.277	0.131	9.752	^*∗∗∗*^
TAD-3 <---LANDSCAPE analysis	1.586	0.157	10.095	^*∗∗∗*^
TAD-2 <---LANDSCAPE analysis	1.139	0.134	8.502	^*∗∗∗*^
TAD-1 <---LANDSCAPE analysis	1.579	0.153	10.328	^*∗∗∗*^
Essential service dept for eco-tourism < ---URBAN PARK _SCAPE	0.233	0.057	4.084	^*∗∗∗*^
Essential service dept for eco-tourism < ---URBAN PARK _SCAPE_001	0.670	0.298	2.251	0.024
Essential service dept for eco-tourism < ---URBAN PARK	−0.051	0.152	−0.333	0.739
Essential service dept for eco-tourism < ---LANDSCAPE analysis	1.050	0.185	5.688	^*∗∗∗*^

**Table 2:** Results comparison.

Models		LVQ [5]	ANN [6]	Deep ML [7]	Deep GA [7]	EST [30]	ANN_LVQ proposed
MATLAB	Accuracy	77.877	83.8687	87.6	84.3035	87.77	88.386
	Specificity	77.7373	83.743	83.7	83.8737	87.37	85.37
	Sensitivity	57.6473	74.43	87.77	87.3456	87.57	88.37

Theory	Accuracy	87.3374	83.76	83.45	83.6433	87.737	88.43
	Specificity	83.7378	83.56	83.7	83.874	85.74	86.37
	Sensitivity	87.6557	87.7	87.3	83	86.84	87.33

## Data Availability

No data were used to support this study.
